# Dynamical Analysis on a Malaria Model with Relapse Preventive Treatment and Saturated Fumigation

**DOI:** 10.1155/2022/1135452

**Published:** 2022-06-28

**Authors:** Dipo Aldila

**Affiliations:** Department of Mathematics, Universitas Indonesia, Depok 16424, Indonesia

## Abstract

Malaria has produced health issues in many parts of the world. One of the reason is due to the recurrence phenomenon, which can happen years after the main infection has appeared in the human body. Furthermore, the fumigation intervention, which has become a major worry in several regions of the world, has yielded unsatisfactory results, as seen by the high number of cases reported each year in several African countries. We present a novel mathematical model that integrates tafenoquine treatments to prevent relapse in the human population and saturation fumigation to control mosquito populations in this study. The endemic threshold, also known as the basic reproduction number, is calculated analytically, as is the existence and local stability of the equilibrium points. Through careful investigation, we discovered that the malaria-free equilibrium is locally asymptotically stable if the basic reproduction number is less than one and unstable if it is greater than one. According to the sensitivity analysis, the utilization of tafenoquine treatment is inversely proportional to the basic reproduction number. Although our model never exhibits a backward bifurcation at the basic reproduction number equal to one, we have demonstrated that it is possible; when the basic reproduction number is greater than one, two stable malaria-endemic equilibrium can exist. As a result, when the basic reproduction number is more than one, the final state will be determined by the initial condition of the population. As a result, enormous temporal fumigation can shift the stability of our malaria model from a big endemic size to a smaller endemic size, which is more advantageous in terms of the malaria prevention strategy. Despite the fact that this is not a case study, the numerical results presented in this article are intended to support any theoretical analysis of current malaria eradication tactics in the field.

## 1. Introduction

Malaria is a vector-borne disease caused by the bite of a female mosquito that has been infected with Plasmodium. Of more than 100 species, only five Plasmodium species cause malaria, namely, Plasmodium vivax, Plasmodium malaria, Plasmodium falciparum, Plasmodium knowlesi, and Plasmodium ovale [1]. When this Plasmodium has entered the human bloodstream, it will attack several vital organs in the human body, especially the liver and red blood cells [2]. People who have been infected with malaria will show a variety of symptoms, including chills, fever, and headache, which can even result in death in most cases in the pediatric population.

Until now, there have been many interventions launched by governments in various countries in the world to tackle the spread of malaria. These interventions include the use of vaccines, treatment, use of insecticide-treated bed nets (ITN), and vector control with fumigation and larvicides [3]. Among these mentioned interventions, vector control with fumigation is considered as the most promising and easiest policy to implement [1]. However, several problems in its implementation arise, such as the tendency of mosquitoes to become resistant to fumigants when the intervention is not well controlled [4] or the problem of limited implementation costs. In some cases in the field, the high fumigation intensity needs to be reduced when infected people are too high. This is due to the difficulty of implementation in the field when intervention costs must also be allocated to treatment for infected individuals in the hospitals.

Vaccines for malaria have become one of the main concerns of governments in many parts of the world and the World Health Organization [5]. In 2021, the R21/Matrix-M vaccine has been investigated to be the second malaria vaccine, and it is stated that it has reached the minimum efficacy limit required by WHO, which is a minimum efficacy of 75% [6]. This type of vaccine has an efficacy level of 77% to reduce the chance of successful infection in humans due to an infected female Anopheles mosquito bite. In addition to vaccination, treatment interventions are also needed to prevent the severity or incidence of relapse in malaria patients. Until now, it was stated that *primaquine* was the primary drug used to avoid relapse in individuals infected with malaria. However, because this drug has to be taken on a regular basis (every 14 days), it has resulted in many treatments not being successful [7]. Therefore, MMV and GlaxoSmithKline (GSK) collaborated to develop a new malaria drug known as *tafenoquine*, which is a single dose treatment for preventing relapse in malaria-infected individuals [8].

The complexity of malaria has attracted the attention of many researchers to take part in efforts to understand the mechanism of spread and the best intervention for malaria. This is due to the complexity of its infection mechanism, such as recurrence phenomena (relapse, reinfection, and recrudescence), to the problem of the most appropriate intervention. Among these researches, mathematical modeling would play an essential role. Many authors have introduced mathematical models to understand how malaria spreads among human and mosquito populations. The first mathematical model for malaria was introduced by Ross in the early 19^th^ century [9], where he introduced the mechanism of malaria transmission involving mosquito and human populations in his model. Ross' research was then continued by Macdonald [10] where he introduced the concept of basic reproduction number in his model. Since then, many mathematical models have been introduced by researchers to understand various important factors in the spread of malaria. Authors in [11] proposed a malaria model considering immunological memory which boost protection of reinfection phenomenon. Two host types in malaria transmission are discussed by author in [12]. Furthermore, a two-age class model for malaria transmission is discussed in [13]. A periodic biting rate of malaria mosquitoes is modelled by author in [14]. They used Floquet theory to analyze the stability of their model. Recently, author in [15] proposed a malaria model with optimal control on saturated treatment rate. Another new strategy of transmission blocking drugs for malaria is modelled by Wu and Hu in [16]. They found that increasing the transmission blocking drugs is a more pronounced effect compared to treatment intervention. Another important factors have been discussed through mathematical models such as vector-bias effect [15, 17], relapse [18, 19], reinfection [20, 21], fumigation [15, 22], temperature and seasonality [23–25], impact of Wolbachia [26], and coinfection [27]. However, the best that we know, there is no mathematical model considering the impact of potential new treatment (tafenoquine) into their model.

In this paper, we introduce and investigate a new mathematical model on malaria transmission. In this model, we divide the human population into five epidemiological classes based on their health status while the mosquito population into two epidemiological classes. Several vital factors were introduced into our model: the effect of a potential new treatment for malaria to prevent relapse; vector-bias phenomena where mosquitoes are more attracted to bite the infected individuals; and fumigation intervention which depends on the number of infected individuals at time *t*. We perform our mathematical analysis to show the existence of a forward bifurcation and forward hysteresis phenomena on our model, which allows the possibility of existence of three different endemic equilibrium, where two of them is locally stable. Based on this phenomenon, we show from a numerical simulation that a massive fumigation intervention in a limited time window can change the dynamic direction of the system from a large endemic equilibrium to a smaller endemic point. We also show a sensitivity analysis to determine the most influential parameter to our model.

This paper is organized as follows. We formulate our model in Section 2. The stability of the malaria-free equilibrium point and the form of the respected basic reproduction number are shown in Section 3. In Section 4, we analyze the existence of the malaria-endemic equilibrium point. In addition, we show the possible forward hysteresis from our model in this section. Some numerical experiments on the proposed model are shown in Section 5. Finally, some relevant conclusions are given in the last section.

## 2. Mathematical Model Formulation

The proposed dynamic model for malaria transmission in this article is inspired by our previous work in [15], by taking into account two important factors. The first factor involved in our new model is the involvement of a malaria relapse prevention drug intervention (for example, tafenoquine [28]). The second factor involves fumigation intervention which is not a monotonous function. We assume that when the number of humans infected with malaria is approaching the outbreak, the intervention given can be quite large. However, when the number of infected people continues to grow, efforts for fumigation will be reduced because of the difficulty of intervention during the outbreak.

This model divides the human population based on their health status and whether they received any malaria treatment or not. Hence, let human population be divided into five epidemiological classes: susceptible (*S*), latent (*E*), infected (*I*), exposed treated (*T*), and recovered (*R*). On the other hand, we classify mosquito population only into two classes: susceptible (*U*) and infected (*W*). The latent individual is an individual who has already been exposed to malaria and has Plasmodium in their lever. If an individual in *E* gets treated with tafenoquine to prevent relapse, then they will be classified into the class of *T*. Only infected individual (*I*) can transmit the Plasmodium into the susceptible mosquito. Based on this assumption, we have the total human population which is given by

(1) $$\begin{array}{c} N_{h}=S+E+T+I+R, \end{array}$$

and the total mosquito population is given by

(2) $$\begin{array}{c} N_{v}=U+W. \end{array}$$

The malaria model is governed by the following system of ordinary differential equations:

(3) $$\begin{array}{c} \frac{dS}{dt}=\Lambda_{h}-\Pi_{h}\left(N,W\right)-\mu_{h}S+\xi R,\\ \frac{dE}{dt}=\Pi_{h}\left(N,W\right)-\left(u_{1}+\eta +\mu_{h}\right)E,\\ \frac{dT}{dt}=u_{1}E-\left(\left(1-p\right)\delta +p\kappa +\mu_{h}\right)T,\\ \frac{dI}{dt}=\left(1-p\right)\delta T+\eta E-\left(\gamma +\mu_{h}\right)I,\\ \frac{dR}{dt}=p\kappa T+\gamma I-\left(\mu_{h}+\xi \right)R,\\ \frac{dU}{dt}=\Lambda_{v}-\Pi_{v}\left(N,U\right)-\left(\mu_{v}+\Psi \left(I,u_{2}\right)\right)U,\\ \frac{dW}{dt}=\Pi_{v}\left(N,U\right)-\left(\mu_{v}+\Psi \left(I,u_{2}\right)\right)W, \end{array}$$

where *Π*_*h*_(*N*, *W*) and *Π*_*v*_(*N*, *U*) are the infection rate in human and mosquito population, respectively, while Ψ(*I*, *u*_2_) presents the fumigation effectiveness factors.

The per capita of birth on humans and mosquitoes is denoted by *Λ*_*h*_ and *Λ*_*v*_, respectively. The natural death rate of humans and mosquitoes is given by *μ*_*h*_ and *μ*_*v*_, respectively. Furthermore, parameters *u*_1_ and *u*_2_ present medical treatment intervention with tafenoquine and vector control with fumigation, respectively. Let*p*be the proportion of exposed individuals who get tafenoquine and succeeded in avoiding relapse after*κ*^−1^duration of treatment. On the other hand, we assume that the 1 − *p* proportion of individuals in *T* failed in treatment. Hence, we have (1 − *p*)*δT* as the transition from *T* to *I* due to treatment failure, where *δ*^−1^ is the incubation period of Plasmodium with the effect of tafenoquine. We denote that the recovery rate from malaria is *γ*, while *ξ*^−1^ is the duration of temporal immunity.

We construct the force of infection in human (*Π*_*h*_(*N*, *W*)) as follows. Let *b* be the average bite per mosquito per day. In our model, we take into account the preference of mosquito to be more attracted to bite infected human, rather than noninfected human. This phenomenon is commonly known as “vector-bias” phenomenon [29]. Based on this “vector-biased” assumption, the probability of a mosquito encountering a susceptible human is given by *S*/(*S* + *E* + *T* + *αI* + *R*), where *α* > 1 is the vector-bias parameter. Hence, total bite of all mosquito per day is given by *bW*(*S*/(*S* + *E* + *T* + *αI* + *R*)). Assuming *ν*_*h*_ as the probability that the bite of infected mosquito succeeded in infecting susceptible human, then *bν*_*h*_*W*(*S*/(*S* + *E* + *T* + *αI* + *R*)) present the total of susceptible human who get infected by malaria per time. Since *b* and *ν*_*h*_ are constant parameters with a dimension of bite/day and 1/(bite × mosquito), respectively, we assume *β*_*h*_≔*bν*_*h*_. Therefore, we have that

(4) $$\begin{array}{c} \Pi_{h}\left(N,W\right)=\beta_{h}W\frac{S}{S+E+T+\alpha I+R}. \end{array}$$

Using a similar approach, let *ν*_*v*_ be the probability of successful infection in mosquitoes; the force of infection on mosquitoes is given by

(5) $$\begin{array}{c} \Pi_{v}\left(N,U\right)=\beta_{v}U\frac{\alpha I}{S+E+T+\alpha I+R}, \end{array}$$

where *β*_*v*_≔*bν*_*v*_ with a dimension of bite/day and 1/(bite × human) for *b* and *ν*_*v*_, respectively.

Now, we construct our fumigation term Ψ(*I*, *u*_2_). We assume that the fumigation intervention depends on the number of infected individuals. Indicators of the endemic of malaria in the field can not be seen from the number of infected mosquitoes, but it can be identified by the high number of infected individuals which is reported in the media. When the number of infected individuals increases, then the intensity of fumigation will increase. However, when the number of infected individuals increases more significantly, then the effectiveness of fumigation will decrease since the policymaker may concentrate more on the number of infected individuals in the hospital, which makes them overwhelmed to control vector population in the field. Hence, we assume that Ψ(*I*, *u*_2_) should have the following properties:

- When the number of the infected individual is zero, then the fumigation intervention is zero. Hence, we have Ψ(0, *u*_2_) = 0
- The fumigation intervention increases at the beginning when the number of infected individual start to increase but will decrease when the number of infected individual is sufficiently large. Hence, we have that ((*∂*Ψ(*I*, *u*_2_))/*∂I*) > 0 for *I* ∈ (0, *I*^critical^) and ((*∂*Ψ(*I*, *u*_2_))/*∂I*) ≤ 0 for *I* ∈ [*I*^critical^, ∞). Note that *I*^critical^ denote the critical number of *I* when the policymaker is already overwhelmed to conduct an effective fumigation intervention in the field

Based on the above assumption, we model our fumigation intervention as

(6) $$\begin{array}{c} \Psi \left(I,u_{2}\right)=u_{2}\frac{I}{a+I^{2}}, \end{array}$$

where *a* > 0 is the saturated coefficient.

According to the mentioned assumptions on the infection and fumigation functions, system (3) now is read as

(7) $$\begin{array}{c} \frac{dS}{dt}=\Lambda_{h}-\beta_{h}W\frac{S}{S+E+T+\alpha I+R}-\mu_{h}S+\xi R,\\ \frac{dE}{dt}=\beta_{h}W\frac{S}{S+E+T+\alpha I+R}-\left(u_{1}+\eta +\mu_{h}\right)E,\\ \frac{dT}{dt}=u_{1}E-\left(\left(1-p\right)\delta +p\kappa +\mu_{h}\right)T,\\ \frac{dI}{dt}=\left(1-p\right)\delta T+\eta E-\left(\gamma +\mu_{h}\right)I,\\ \frac{dR}{dt}=p\kappa T+\gamma I-\left(\mu_{h}+\xi \right)R,\\ \frac{dU}{dt}=\Lambda_{v}-\beta_{v}U\frac{\alpha I}{S+E+T+\alpha I+R}-\left(\mu_{v}+u_{2}\frac{I}{a+I^{2}}\right)U,\\ \frac{dW}{dt}=\beta_{v}U\frac{\alpha I}{S+E+T+\alpha I+R}-\left(\mu_{v}+u_{2}\frac{I}{a+I^{2}}\right)W, \end{array}$$

with a nonnegative initial conditions given at time *t* = 0.  Figure 1 depicts the flow chart of our malaria transmission model. Biological interpretation and the unity of all parameters in system (7) are given in Table 1.

Let system (7) have an initial condition in the following set:

(8) $$\begin{array}{c} D=\left\{\left(S,E,T,I,R,U,W\right)\in {\mathbb{R}}_{+}^{7}\left|S,U>0,E,T,I,R,W\geq 0\right.\right\}. \end{array}$$

To describe the feasible solution of system (7) and its biological interpretation, we have the following theorem.

**Theorem 1 .**

For initial values in (8), malaria model in system (7) has a unique solution and remains in *𝒟* for all time *t* ≥ 0.

**Proof**

Please see Appendix A for the proof.

## 3. Malaria-Free Equilibrium and the Basic Reproduction Number

The first equilibrium point of our model is the malaria-free equilibrium point. This equilibrium present a situation where all nonsusceptible population do not exist in the equilibrium condition. For this reason, let *E* = 0, *T* = 0, *I* = 0, *R* = 0, and *W* = 0, and then, malaria-free equilibrium (*MFE*) is obtained by the following subsystem:

(9) $$\begin{array}{c} \frac{dS}{dt}=\Lambda_{h}-\mu_{h}S,\\ \frac{dU}{dt}=\Lambda_{v}-\mu_{v}U. \end{array}$$

Taking the right hand side of the above system, it follows that the malaria-free equilibrium of system (7) is given by

(10) $$\begin{array}{c} MFE=\left(S^{*},E^{*},T^{*},I^{*},R^{*},U^{*},W^{*}\right)=\left(\frac{\Lambda_{h}}{\mu_{h}},0,0,0,0,\frac{\Lambda_{v}}{\mu_{v}},0\right). \end{array}$$

To conduct further analysis on the qualitative behaviour of our model, it is important to determine the related basic reproduction number of our proposed model. In many epidemiological models, basic reproduction number holds an important role in determining that the diseases die out or exist in the population [34–38]. Basic reproduction number is defined as the expected number of secondary cases caused by one primary case during infection period in a completely susceptible population [39, 40]. The basic reproduction number is calculated using the next-generation matrix approach [41]. From system (7), we have that the infected compartments consist of *E*, *T*, *I*, and *W*. The Jacobian matrix of subsystem of infected compartment on system (7) evaluated in *MFE* can be written as *ℱ* + *𝒱*, where

(11) $$\begin{array}{c} F=\left[\begin{array}{cccc} 0 & 0 & 0 & \beta_{h}\\ 0 & 0 & 0 & 0\\ 0 & 0 & 0 & 0\\ 0 & 0 & \frac{\beta_{v}\Lambda_{v}\alpha \;\mu_{h}}{\mu_{v}\Lambda_{h}} & 0 \end{array}\right],\\ V=\left[\begin{array}{cccc} -u_{1}-\eta -\mu_{h} & 0 & 0 & 0\\ u_{1} & -\left(1-p\right)\delta -\kappa \;p-\mu_{h} & 0 & 0\\ \eta & \left(1-p\right)\delta & -\gamma -\mu_{h} & 0\\ 0 & 0 & 0 & -\mu_{v} \end{array}\right], \end{array}$$

where *ℱ* and *𝒱* present the transmission and transition terms. Using formula in [41], we have the next-generation matrix (*NGM*) of system (7) which is given by

(12) $$\begin{array}{c} NGM=-E^{T}FV^{-1}E=\left[\begin{array}{cc} 0 & \frac{\beta_{h}}{\mu_{v}}\\ \frac{\alpha \;\Lambda_{v}\beta_{v}\mu_{h}\left(\delta \;\eta \;p+\delta \;pu_{1}-\eta \;\kappa \;p-\delta \;\eta -\delta \;u_{1}-\eta \;\mu_{h}\right)}{\mu_{v}\Lambda_{h}\left(u_{1}+\eta +\mu_{h}\right)\left(\delta \;p-\kappa \;p-\delta -\mu_{h}\right)\left(\gamma +\mu_{h}\right)} & 0 \end{array}\right], \end{array}$$

where *E*^*T*^ is the transpose of *E*, with

(13) $$\begin{array}{c} E=\left[\begin{array}{cc} 1 & 0\\ 0 & 0\\ 0 & 0\\ 0 & 1 \end{array}\right]. \end{array}$$

Note that each column of *ℱ* can be spanned by each column of *E*. Hence, the basic reproduction number of system (7) is given by

(14) $$\begin{array}{c} R_{0}=\sqrt{\frac{\beta_{v}\Lambda_{v}\alpha \;\mu_{h}\left(\delta \left(\eta +u_{1}\right)\left(1-p\right)+\eta \left(\mu_{h}+p\kappa \right)\right)\beta_{h}}{\Lambda_{h}{\mu_{v}}^{2}\left(\delta \left(1-p\right)+\mu_{h}+p\kappa \right)\left(u_{1}+\eta +\mu_{h}\right)\left(\gamma +\mu_{h}\right)}}. \end{array}$$

More example on the method of next-generation matrix method to determine the basic reproduction number in various epidemiological models can be seen in [42–44]. The above expression can be rewritten as a multiplication between four important component on malaria transmission on system (7) as follows.

(15) $$\begin{array}{c} R_{0}=\sqrt{C_{1}\times C_{2}\times C_{3}\times C_{4}}, \end{array}$$

where *𝒞*_1_ = *β*_*h*_/(*u*_1_ + *η* + *μ*_*h*_) present the number of new latent infected human per infection period of *E*, *𝒞*_2_ = *αβ*_*v*_/*μ*_*v*_ present the number of new infected mosquitoes per infection period of *W*, *𝒞*_3_ = *N*_*v*_/*N*_*h*_ present the ratio of mosquitoes and human, and *𝒞*_4_ = *η* + *u*_1_(1/(1 + ((*pκ* + *μ*_*h*_)/((1 − *p*)*δ*)))) present the impact of tafenoquine intervention.

According to Theorem 2 in [45], we have the following theorem regarding the local stability criteria of the malaria-free equilibrium of system (7).

**Theorem 2 .**

The malaria-free equilibrium of system (7) is locally asymptotically stable if *ℛ*_0_ < 1 and unstable if *ℛ*_0_ > 1.

### 3.1. Sensitivity Analysis on the Basic Reproduction Number

In many mathematical epidemiology models, understanding the impact of key parameters in determining the size of the basic reproduction number is essential to find the best optimal strategy. Therefore, we study the normalized sensitivity analysis of the basic reproduction number using the following formula [30]:

(16) $$\begin{array}{c} \Gamma_{\rho }^{R_{0}}=\frac{\partial R_{0}}{\partial p}\times \frac{p}{R_{0}}, \end{array}$$

where *ρ* is any key parameter in malaria model in system (7). In our paper, we are only interested in the following parameters: *β*_*h*_, *β*_*v*_, *α*, *u*_1_, *u*_2_, *η*, *δ*, *p*, *κ*, *γ*, *ξ*, and *a*. Furthermore, we do not show the partial derivative of these parameters since it has a long expressions. Using parameter values as in Table 1, *u*_1_ = 0.2, *u*_2_ = 0, and *p* = 0.8; the normalized sensitivity of *ℛ*_0_ is given in Table 2 and visualized in Figure 2.

The normalized indices in Table 2 are a nondimensional value, which present the percentage change of *ℛ*_0_ for each increase value of parameter *ρ* for 1%. For an example, since Γ_*p*_^*ℛ*_0_^ = −0.6477, then increasing probability of individuals in *T* to succeed in treatment for 10% will reduce *ℛ*_0_ for 6.477%. On the other hand, since Γ_*β*_*h*__^*ℛ*_0_^ = 0.5, then increasing *β*_*h*_ for 10% will increase *ℛ*_0_ for 5%. From Figure 2, we can see that *β*_*h*_, *β*_*v*_, *α*, *η*, and *δ* are proportional to *ℛ*_0_. Increasing these mentioned values will increase *ℛ*_0_. On the other hand, parameters *p*, *γ*, *u*_1_, and *κ* are inversely proportional to *ℛ*_0_. Therefore, increasing the value of *p*, *γ*, *u*_1_, and *κ* will reduce *ℛ*_0_. In addition, we can see that fumigation (*u*_2_), rate of loss of immunity (*ξ*), and saturated parameter (*a*) do not affect *ℛ*_0_. Figure 2 shows the most to the less influential parameter to *ℛ*_0_ in descending order, from left to the right.

Figure 3 shows the level set of *ℛ*_0_ with respect to *u*_1_, *α*, and *p*. From Figure 3(a), we can see that increasing the value of *p* reduces *ℛ*_0_. It means that more people succeed due to treatment with tafenoquine; then, the possibility to achieve malaria-free equilibrium is bigger. Same interpretation to the rate of treatment *u*_1_. We can see that more intense intervention of tafenoquine will reduce *ℛ*_0_. In addition, we can see clearly that better quality of tafenoquine will reduce the burden of intervention in providing tafenoquine treatment to achieve malaria-free conditions. The effect of vector-bias on the success of tafenoquine intervention to reduce *ℛ*_0_ can be seen in Figure 3(b). We can see that more bias the mosquito to be more preferring infected human will increase the *ℛ*_0_, which makes the intervention of tafenoquine should be given more intense to reduce the value of *ℛ*_0_.

## 4. The Malaria-Endemic Equilibrium

### 4.1. Existence of Malaria-Endemic Equilibrium

The malaria-endemic equilibrium of system (7) is given by

(17) $$\begin{array}{c} MEE=\left(S^{†},E^{†},T^{†},I^{†},R^{†},U^{†},W^{†}\right), \end{array}$$

where

(18) $$\begin{array}{c} S^{†}=\frac{\Lambda_{h}}{\mu_{h}}-E^{†}-I^{†}-T^{†}-R^{†},\\ E^{†}=\frac{I^{†}\left(\delta \left(\mu_{h}+\gamma \right)\left(1-p\right)+\left(\gamma +\mu_{h}\right)\left(\mu_{h}+p\kappa \right)\right)}{\delta \left(u_{1}+\eta \right)\left(1-p\right)+\eta \left(\mu_{h}+p\kappa \right)},\\ T^{†}=\frac{I^{†}u_{1}\left(\gamma +\mu_{h}\right)}{\delta \left(u_{1}+\eta \right)\left(1-p\right)+\eta \left(\mu_{h}+p\kappa \right)},\\ R^{†}=\frac{\left(\delta \left(\gamma +\mu_{h}\right)\left(1-p\right)+\gamma \kappa p\left(\eta +\mu_{h}\right)+\mu_{h}\left(\eta \gamma +p\kappa u_{1}\right)\right)}{\left(\delta \left(u_{1}+\eta \right)\left(1-p\right)+\eta \left(\mu_{h}+p\kappa \right)\right)\left(\xi +\mu_{h}\right)},\\ U^{†}=\frac{\Lambda_{v}\left(S^{†}+E^{†}+\alpha I^{†}+T^{†}+R^{†}\right)\left(a+{\left(I^{†}\right)}^{2}\right)}{\Sigma_{i=0}^{3}c_{i}},\\ W^{†}=\frac{\Lambda_{v}\left(a+{\left(I^{†}\right)}^{2}\right)}{\left(u_{2}I^{†}\right)+\mu_{v}\left(a+{\left(I^{†}\right)}^{2}\right)}-U^{†}, \end{array}$$

with *c*_0_ = *αμ*_*v*_(*S*^†^ + *E*^†^ + *T*^†^ + *R*^†^), *c*_1_ = *aα*(*β*_*v*_ + *μ*_*v*_) + *u*_2_(*S*^†^ + *E*^†^ + *T*^†^ + *R*^†^), *c*_2_ = *αu*_2_ + *μ*_*v*_(*S*^†^ + *E*^†^ + *T*^†^ + *R*^†^), and *c*_3_ = *α*(*β*_*v*_ + *μ*_*v*_). Note that *I*^†^ is taken from the positive root of the following polynomial:

(19) $$\begin{array}{c} G\left(\Omega ,I\right)=\overset{6}{\underset{j=1}{\sum }}k_{j}I^{j}=0, \end{array}$$

where *Ω* is the set of parameter in system (7), and

(20) $$\begin{array}{c} k_{6}=-\mu_{h}^{2}\mu_{v}\left(\xi +\mu_{h}\right)\left(\delta \left(1-p\right)+\mu_{h}+p\kappa \right)\left(\alpha -1\right)\left(u_{1}+\eta +\mu_{h}\right)\left(\alpha \beta_{v}+\mu_{v}\left(\alpha -1\right)\right)\left(\gamma +\mu_{h}\right),\\ k_{0}=\Lambda_{h}{\mu_{v}}^{2}\left(\delta \left(1-p\right)+\mu_{h}+p\kappa \right)\left(u_{1}+\eta +\mu_{h}\right)\left(\gamma +\mu_{h}\right)\left(R_{0}^{2}-1\right), \end{array}$$

while *k*_5_, *k*_4_, *k*_3_, *k*_2_, and *k*_1_ have a complex form to be written in this article. It can be seen that whenever *I*^†^ > 0, then *E*^†^, *T*^†^, *R*^†^, and *U*^†^ are also positive. On the other hand, *S*^†^ is always positive since *N*_*h*_ ≤ (*Λ*_*h*_/*μ*_*h*_) (see the proof of Theorem 1). On the other hand, since

(21) $$\begin{array}{c} W^{†}=\frac{\Lambda_{v}\left(a+{\left(I^{†}\right)}^{2}\right)}{\left(u_{2}I^{†}\right)+\mu_{v}\left(a+{\left(I^{†}\right)}^{2}\right)}-U^{†}<\frac{\Lambda_{v}}{\mu_{v}}-U^{†} \end{array}$$

and *N*_*v*_ ≤ (*Λ*_*v*_/*μ*_*v*_) (see the proof of Theorem 1), then we can guarantee that *W*^†^ is also positive.

From the expression of polynomial in (19), *k*_6_ is always negative since *α* > 1, *k*_0_ > 0 ⇐ *ℛ*_0_ > 1, while another coefficient is difficult to be determined, whether it was positive or negative. Hence, using the Descartes rules of sign [46], there exists at least one positive root of polynomial (19) whenever *ℛ*_0_ > 1. According to this result and the expression of *MEE*, we have the following result.

**Theorem 3 .**

System (7) has at least one malaria-endemic equilibrium point if *ℛ*_0_ > 1.

Since polynomial in (19) is a six-degree polynomial, it is possible that system (7) have more than one malaria-endemic equilibrium point. We use Descartes rules of sign [46] to analyze the maximum possibility of positive root of polynomial in (19). The result is given in Table 3 for the case when *ℛ*_0_ > 1, and Table 4 for the case when *ℛ*_0_ < 1.

From Table 2, we can confirm the result in Theorem 3 that we always have at least one malaria-endemic equilibrium when *ℛ*_0_ > 1. If *ℛ*_0_ > 1, then we always have an odd number possibility of the positive root of polynomial (19), i.e., 1, 3, or 5 positive roots. On the other hand, malaria-endemic equilibrium is possible to vanish only when *ℛ*_0_ < 1. However, we still possible to have 2, 4, or 6 positive roots of polynomial (19) when *ℛ*_0_ < 1.

### 4.2. Bifurcation Analysis

In this section, we perform the bifurcation analysis of our proposed malaria model in system (7). To do this analysis, we use the well-known Castillo-Song bifurcation theorem [47] (please see [48–51] for more examples on the use of this theorem on epidemiological models). First, for numerical calculation purposes, let us redefine our proposed system (7) as follows:

(22) $$\begin{array}{c} f_{1}≔\Lambda_{h}-\beta_{h}x_{6}\frac{x_{1}}{x_{1}+x_{2}+x_{3}+\alpha x_{4}+x_{5}}-\mu_{h}x_{1}+\xi x_{5},\\ f_{2}≔\beta_{h}x_{6}\frac{x_{1}}{x_{1}+x_{2}+x_{3}+\alpha x_{4}+x_{5}}-\left(u_{1}+\eta +\mu_{h}\right)x_{2},\\ f_{3}≔u_{1}x_{2}-\left(\left(1-p\right)\delta +p\kappa +\mu_{h}\right)x_{3},\\ f_{4}≔\left(1-p\right)\delta x_{3}+\eta x_{2}-\left(\gamma +\mu_{h}\right)x_{4},\\ f_{5}≔p\kappa x_{3}+\gamma x_{4}-\left(\mu_{h}+\xi \right)x_{5},\\ f_{6}≔\Lambda_{v}-\beta_{v}x_{6}\frac{\alpha x_{4}}{x_{1}+x_{2}+x_{3}+\alpha x_{4}+x_{5}}-\left(\mu_{v}+u_{2}\frac{x_{4}}{a+x_{4}^{2}}\right)x_{6},\\ f_{7}≔\beta_{v}x_{6}\frac{\alpha x_{4}}{x_{1}+x_{2}+x_{3}+\alpha x_{4}+x_{5}}-\left(\mu_{v}+u_{2}\frac{x_{4}}{a+x_{4}^{2}}\right)x_{7}, \end{array}$$

where *x*_*i*_ for *i* = 1, 2, ⋯7 present *S*, *E*, *T*, *I*, *R*, *U*, and *W*, respectively, Next, we determine our bifurcation parameter to replace *ℛ*_0_. By solving *ℛ*_0_ = 1 with respect to *β*_*h*_, we obtain the bifurcation parameter, namely, *β*_*h*_ = *β*^∗^, as follows:

(23) $$\begin{array}{c} \beta_{h}=\beta^{*}=\frac{\left(\left(p-1\right)\delta -\kappa \;p-\mu_{h}\right)\left(\gamma +\mu_{h}\right)\left(u_{1}+\eta +\mu_{h}\right){\mu_{v}}^{2}\Lambda_{h}}{\left(\left(u_{1}+\eta \right)\left(p-1\right)\delta -\eta \;\left(\kappa \;p+\mu_{h}\right)\right)\mu_{h}\beta_{v}\alpha \;\Lambda_{v}}. \end{array}$$

The linearization of *MFE* of system (22) at *β*_*h*_ = *β*^∗^ is given by

(24) $$\begin{array}{c} {\left.J\right|}_{MFE}≔\left[\begin{array}{ccccccc} -\mu_{h} & 0 & 0 & 0 & \xi & 0 & c_{17}\\ 0 & c_{22} & 0 & 0 & 0 & 0 & c_{27}\\ 0 & u_{1} & c_{33} & 0 & 0 & 0 & 0\\ 0 & \eta & \left(1-p\right)\delta & -\gamma -\mu_{h} & 0 & 0 & 0\\ 0 & 0 & \kappa \;p & \gamma & -\xi -\mu_{h} & 0 & 0\\ 0 & 0 & 0 & c_{64} & 0 & -\mu_{v} & 0\\ 0 & 0 & 0 & \frac{\beta_{v}\Lambda_{v}\alpha \;\mu_{h}}{\mu_{v}\Lambda_{h}} & 0 & 0 & -\mu_{v} \end{array}\right], \end{array}$$

with

(25) $$\begin{array}{c} c_{17}=-\frac{\left(\left(p-1\right)\delta -\kappa \;p-\mu_{h}\right)\left(\gamma +\mu_{h}\right)\left(u_{1}+\eta +\mu_{h}\right){\mu_{v}}^{2}\Lambda_{h}}{\left(\left(u_{1}+\eta \right)\left(p-1\right)\delta -\eta \;\left(\kappa \;p+\mu_{h}\right)\right)\mu_{h}\beta_{v}\alpha \;\Lambda_{v}},\\ c_{22}=-u_{1}-\eta -\mu_{h},\\ c_{27}=\frac{\left(\left(p-1\right)\delta -\kappa \;p-\mu_{h}\right)\left(\gamma +\mu_{h}\right)\left(u_{1}+\eta +\mu_{h}\right){\mu_{v}}^{2}\Lambda_{h}}{\left(\left(u_{1}+\eta \right)\left(p-1\right)\delta -\eta \;\left(\kappa \;p+\mu_{h}\right)\right)\mu_{h}\beta_{v}\alpha \;\Lambda_{v}},\\ c_{33}=-\left(1-p\right)\delta -\kappa \;p-\mu_{h},\\ c_{64}=-\frac{\beta_{v}\Lambda_{v}\alpha \;\mu_{h}}{\mu_{v}\Lambda_{h}}-\frac{u_{2}\Lambda_{v}}{a\mu_{v}}. \end{array}$$

The Jacobian matrix *J*_*MFE*_ has a simple zero eigenvalue, and the other three eigenvalues are explicitly negative (−*μ*_*h*_, −*μ*_*h*_, −(*μ*_*h*_ + *ξ*)), while the other three is coming from the root of the following polynomial:

(26) $$\begin{array}{c} P\left(\lambda \right)=c_{3}\lambda^{3}+c_{2}\lambda^{2}+c_{1}\lambda +c_{0}=0, \end{array}$$

where

(27) $$\begin{array}{c} c_{3}=\Lambda_{h}\mu_{v}\left(u_{1}+\mu_{v}+3\mu_{h}+\eta +\gamma +p\kappa +\delta \left(1-p\right)\right),\\ c_{2}=\delta \left(1-p\right)\left(\eta +\gamma +u_{1}+\mu_{v}+2\mu_{h}\right)\left(3\mu_{h}^{2}+\mu_{h}\left(2\kappa p+2\eta +2\gamma +3\mu_{v}+2u_{1}\right)+\cdots \right.+\left.\mu_{v}\left(\kappa p+\eta +\gamma +u_{1}\right)+\gamma \left(\kappa p+\eta +u_{1}\right)+p\kappa \left(\eta +u_{1}\right)\right),\\ c_{1}=\left[\mu_{v}^{2}\left(3\mu_{h}^{2}+\mu_{h}\left(2\left(1-p\right)\delta +2\kappa p+\eta +\gamma +u_{1}\right)+\delta \left(1-p\right)\left(\eta +\gamma +u_{1}\right)+p\kappa \left(\eta +\gamma +u_{1}\right)\right)\right.+\left.\left(\eta +u_{1}+\mu_{h}\right)\left(\left(1-p\right)\delta +p\kappa +\mu_{h}\right)\left(\gamma +\mu_{h}\right)\right]\Lambda_{h}+\Lambda_{v}\alpha \eta \beta^{*}\beta_{v}\mu_{h},\\ c_{0}=\Lambda_{h}\mu_{v}^{2}\left(\gamma +\mu_{h}\right)\left(u_{1}+\eta +\mu_{h}\right)\left(\left(1-p\right)\delta +p\kappa +\mu_{h}\right)+\beta_{h}^{*}\beta_{v}\mu_{h}\alpha \Lambda_{v}\left(\delta \left(1-p\right)\left(\eta +u_{1}\right)+p\kappa \eta +\eta \mu_{h}\right). \end{array}$$

Since (1 − *p*) > 0, then *c*_*i*_ for *i* = 0, 1, 2, 3 are positive. Since all the coefficients of *P*(*λ*) are positive, then all other three eigenvalues of *J*|_*MFE*_ are negative. Therefore, we can continue using the center manifold theory to analyze the bifurcation phenomena at *ℛ*_0_ = 1. Next, we use the Castillo-Chavez and Song theorem [47] to analyze the bifurcation phenomena of system (7) at *ℛ*_0_ = 1.

First, we calculate the right and left eigenvector of *J*|_*MFE*_ with respect to the zero eigenvalue. The right eigenvector is given by **w** = (*w*_1_, *w*_2_, *w*_3_, *w*_4_, *w*_5_, *w*_6_, *w*_7_)^*T*^, with

(28) $$\begin{array}{c} w_{1}=\frac{1}{\left(\gamma +\mu_{h}\right)\left(\xi +\mu_{h}\right)u_{1}}\;\left(-{\mu_{h}}^{3}+\left(\left(p-1\right)\delta -\kappa \;p-\xi -\eta -\gamma -u_{1}\right){\mu_{h}}^{2}+\right.\left(\left(\xi +\eta +\gamma +u_{1}\right)\left(p-1\right)\delta -\kappa \;\left(\xi +\eta +\gamma +u_{1}\right)p+\left(-\xi -\eta -u_{1}\right)\gamma -\xi \;\left(u_{1}+\eta \right)\right)\mu_{h}+\left.\left(p-1\right)\left(\left(\xi +\eta +u_{1}\right)\gamma +\xi \;\left(u_{1}+\eta \right)\right)\delta -\kappa \;\left(\left(\xi +\eta +u_{1}\right)\gamma +\eta \;\xi \right)p-\gamma \;\xi \;u_{1}\right),\\ w_{2}=-\frac{\left(\delta \;p-\kappa \;p-\delta -\mu_{h}\right)}{u_{1}},\\ w_{3}=1,\\ w_{4}=-\frac{\delta \;\eta \;p+\delta \;pu_{1}-\eta \;\kappa \;p-\delta \;\eta -\delta \;u_{1}-\eta \;\mu_{h}}{\left(\gamma +\mu_{h}\right)u_{1}},\\ w_{5}=\frac{\left(\left(\left(-\delta +\kappa \right)p+\delta \right)u_{1}-\eta \;\left(\left(\delta -\kappa \right)p-\delta -\mu_{h}\right)\right)\gamma +\kappa \;p\mu_{h}u_{1}}{\left(\gamma +\mu_{h}\right)\left(\xi +\mu_{h}\right)u_{1}},\\ w_{6}=-\frac{\left(a\alpha \;\beta_{v}\mu_{h}+u_{2}\Lambda_{h}\right)\left(-\left(u_{1}+\eta \right)\left(p-1\right)\delta +\eta \;\left(\kappa \;p+\mu_{h}\right)\right)w3\;\Lambda_{v}}{u_{1}\left(\gamma +\mu_{h}\right)a\Lambda_{h}{\mu_{v}}^{2}},\\ w_{7}=-\frac{\Lambda_{v}\alpha \;\beta_{v}\;\mu_{h}\left(\left(\eta +u_{1}\right)\left(p-1\right)\delta -\eta \;\left(\kappa \;p+\mu_{h}\right)\right)}{\Lambda_{h}{\mu_{v}}^{2}\left(\gamma +\mu_{h}\right)u_{1}}. \end{array}$$

On the other hand, the left eigenvector is given by **v** = (*v*_1_, *v*_2_, *v*_3_, *v*_4_, *v*_5_, *v*_6_, *v*_7_) where

(29) $$\begin{array}{c} v_{1}=0,\\ v_{2}=\frac{\left(\eta +u_{1}\right)\left(p-1\right)\delta -\eta \;\left(\kappa \;p+\mu_{h}\right)}{\left(\eta +u_{1}+\mu_{h}\right)\delta \;\left(p-1\right)},\\ v_{3}=1,\\ v_{4}=\frac{\left(p-1\right)\delta -\kappa \;p-\mu_{h}}{\left(p-1\right)\delta },\\ v_{5}=0,\\ v_{6}=0,\\ v_{7}=\frac{\left(\gamma +\mu_{h}\right)\Lambda_{h}\mu_{v}\left(\left(p-1\right)\delta -\kappa \;p-\mu_{h}\right)}{\Lambda_{v}\alpha \;\beta_{v}\mu_{h}\delta \;\left(p-1\right)}. \end{array}$$

It is obvious that *v*_1_ = *v*_5_ = *v*_6_ = 0. Furthermore, *f*_3_ and *f*_4_ are one degree functions. Thus, we only need to consider the second-order partial derivative of *f*_2_ and *f*_7_. By algebraic computation, we obtain the following second-order partial derivatives which have nonzero values after substituting the *MFE*.

(30) $$\begin{array}{c} \frac{\partial^{2}f_{2}}{\partial x_{2}\partial x_{7}}=\frac{\partial^{2}f_{2}}{\partial x_{7}\partial x_{2}}=-\frac{\beta_{h}\mu_{h}}{\Lambda_{h}},\frac{\partial^{2}f_{2}}{\partial x_{3}\partial x_{7}}=\frac{\partial^{2}f_{2}}{\partial x_{7}\partial x_{3}}=-\frac{\beta_{h}\mu_{h}}{\Lambda_{h}},\\ \frac{\partial^{2}f_{2}}{\partial x_{4}\partial x_{7}}=\frac{\partial^{2}f_{2}}{\partial x_{7}\partial x_{4}}=-\frac{\beta_{h}\mu_{h}\alpha }{\Lambda_{h}},\frac{\partial^{2}f_{2}}{\partial x_{5}\partial x_{7}}=\frac{\partial^{2}f_{2}}{\partial x_{7}\partial x_{5}}=-\frac{\beta_{h}\mu_{h}}{\Lambda_{h}},\\ \frac{\partial^{2}f_{7}}{\partial x_{1}\partial x_{4}}=\frac{\partial^{2}f_{7}}{\partial x_{4}\partial x_{1}}=-\frac{\beta_{v}\Lambda_{v}\alpha \;{\mu_{h}}^{2}}{\mu_{v}{\Lambda_{h}}^{2}},\frac{\partial^{2}f_{7}}{\partial x_{2}\partial x_{4}}=\frac{\partial^{2}f_{7}}{\partial x_{4}\partial x_{2}}=-\frac{\beta_{v}\Lambda_{v}\alpha \;{\mu_{h}}^{2}}{\mu_{v}{\Lambda_{h}}^{2}},\\ \frac{\partial^{2}f_{7}}{\partial x_{3}\partial x_{4}}=\frac{\partial^{2}f_{7}}{\partial x_{4}\partial x_{3}}=-\frac{\beta_{v}\Lambda_{v}\alpha \;{\mu_{h}}^{2}}{\mu_{v}{\Lambda_{h}}^{2}},\frac{\partial^{2}f_{7}}{\partial x_{5}\partial x_{4}}=\frac{\partial^{2}f_{7}}{\partial x_{4}\partial x_{5}}=-\frac{\beta_{v}\Lambda_{v}\alpha \;{\mu_{h}}^{2}}{\mu_{v}{\Lambda_{h}}^{2}},\\ \frac{\partial^{2}f_{7}}{\partial x_{4}\partial x_{6}}=\frac{\partial^{2}f_{7}}{\partial x_{6}\partial x_{4}}=\frac{\beta_{v}\alpha \;\mu_{h}}{\Lambda_{h}},\frac{\partial^{2}f_{7}}{\partial x_{4}\partial x_{7}}=\frac{\partial^{2}f_{7}}{\partial x_{7}\partial x_{4}}=-\frac{u_{2}}{a},\\ \frac{\partial^{2}f_{7}}{\partial x_{4}\partial x_{4}}=-2\;\frac{\beta_{v}\Lambda_{v}\alpha^{2}{\mu_{h}}^{2}}{\mu_{v}{\Lambda_{h}}^{2}}. \end{array}$$

For the bifurcation indicators, we calculate *𝒜* for system (22) which is expressed by

(31) $$\begin{array}{c} A=v_{2}\overset{7}{\underset{i,j=1}{\sum }}w_{i}\frac{\partial^{2}f_{2}}{\partial x_{i}\partial x_{j}}+v_{7}\overset{7}{\underset{i=1}{\sum }}w_{i}\frac{\partial^{2}f_{7}}{\partial x_{i}\partial x_{j}}. \end{array}$$

We can confirm that *𝒜* is always negative (please see the expression of *𝒜* in Appendix D). Meanwhile, *ℬ* is given by

(32) $$\begin{array}{c} B=v_{2}\overset{7}{\underset{i=1}{\sum }}w_{i}\frac{\partial^{2}f_{2}}{\partial x_{i}\partial \beta_{h}}=\frac{{\left(\left(u_{1}+\eta \right)\left(p-1\right)\delta -\eta \;\left(\kappa \;p+\mu_{h}\right)\right)}^{2}\mu_{h}\beta_{v}\alpha \;\Lambda_{v}}{\left(u_{1}+\eta +\mu_{h}\right)\delta \;\left(1-p\right)\Lambda_{h}{\mu_{v}}^{2}\left(\gamma +\mu_{h}\right)u_{1}}. \end{array}$$

Since all parameters are positive, and (1 − *p*) > 0, then we have that *ℬ* > 0. According to Castillo-Chavez and Song theorem [47], since the quantity of *𝒜* is negative and *ℬ* is positive, then system (22)) indicates a forward bifurcation at *ℛ*_0_ = 1. We state the result in the following theorem.

**Theorem 4 .**

System (7) always exhibits a forward bifurcation at *ℛ*_0_ = 1.

### 4.3. Numerical Experiments on Theorem 4

In this section, we show the numerical interpretation of Theorem 4. The first numerical experiment is for the bifurcation diagram of system (7), which is given in Figure 4. We use parameter values as mentioned in Table 1, except that it states differently. With this set of parameter values, we have *ℛ*_0_ = 1 when *β*_*h*_ = 0.0004079. For the case of *a* = 400, *u*_1_ = 0.2, and *u*_2_ = 0, the bifurcation diagram is shown in Figure 4(a). It can be seen that the forward bifurcation phenomenon appears, which indicates there always exists a unique endemic equilibrium point when *ℛ*_0_ > 1, and no endemic equilibrium when *ℛ*_0_ < 1. Furthermore, we can see that the malaria-endemic equilibrium is always stable (solid red) when *ℛ*_0_ > 1. The autonomous simulation for various initial conditions is shown in Figure 5. We use Runge-Kutta adaptive step size method in MATLAB to run the autonomous simulation in this article [52] (please see [53] for further detail on the method and its algorithm). It can be seen that when *ℛ*_0_ = 0.8 < 1, then the solution from all different initial conditions tends to the malaria-free equilibrium point (Figure 5). On the other hand, when *ℛ*_0_ > 1, then all trajectories tend to the malaria-endemic equilibrium (Figure 6).

The autonomous simulation of system (7) when forward hysteresis (Figure 4(b)) appears is given in Figures 7 and 8. The numerical results is using the same parameter values as in Figure 4(b). We only conduct two cases for this scenario, namely, when *ℛ*_0_ > 1 but close to one in which only one stable malaria-endemic appears (Figure 7) and when two stable malaria-endemic equilibrium appears (Figure 8) when *ℛ*_0_ > 1, but not too far from 1. In the first case, as shown in Figure 7, we can see that all trajectories from all different initial conditions tend to the same malaria-endemic equilibrium. However, when hysteresis starts to appear, which causes two stable malaria-endemic equilibrium, the solutions will tend to two different stable malaria-endemic equilibrium points, depending on their initial conditions. We can see that when the initial condition is close enough to the bigger malaria-endemic equilibrium (blue curve), then the solution tends to the bigger size of malaria-endemic equilibrium. The same thing happens when the initial value of infection is small enough, and then, the solution leads to the smallest stable malaria-endemic equilibrium. These simulation results indicate that fumigation may trigger the existence of multiple stable malaria-endemic equilibrium for some value when *ℛ*_0_ > 1.  Figure 9 confirms the statement. It can be seen that an increase in fumigation rate increases the interval when multiple stable malaria-endemic equilibrium appears.

## 5. Autonomous Simulation

From the previous mathematical analysis, we found that our proposed malaria model always exhibits a forward bifurcation at *ℛ*_0_ = 1. These results indicate that the basic reproduction number becomes the only endemic indicator on our proposed model. However, our model may show a multiple stable endemic equilibrium when *ℛ*_0_ > 1. This phenomenon is called a forward hysteresis [54]. We found that this phenomenon was affected by the intensity of fumigation (*u*_2_) and the level of population awareness (*a*). Furthermore, our sensitivity analysis indicates how important is the intervention of tafenoquine to prevent the occurrence of relapse and fumigation to control the number of Anopheles mosquitoes in the environment. To visualize our mentioned results, we perform several numerical simulations on our autonomous simulations for several scenarios.

### 5.1. Effect of Vector-Bias

In malaria transmission, vector-bias has an important role in determining the endemic condition of the population [29]. The larger the vector-bias values, the more mosquito attracted to hunt infected humans for their meal.  Figure 10 depicts the dynamic of the solution of our malaria model in (7) for several values of vector-bias parameter. We use the same parameter values as in Table 2, except *u*_1_ = 0.1, *u*_2_ = 0.05, *p* = 0.8, and varying *α* from 1 to 5. With these parameters, *ℛ*_0_ is always larger than 1, which makes the solution of system (7) tends to the malaria-endemic equilibrium. We can see that an increased value of the vector-bias parameter at the malaria-endemic equilibrium situation will increase the total population in infected humans but reduce the size of the infected mosquito population. This means that the more Anopheles mosquitoes attracted to bite infected humans than healthy humans can negatively impact the human population, where the endemic size can increase. Therefore, efforts to control the mosquito population are essential in this situation.

### 5.2. Effect of Fumigation Saturation Parameter

The first autonomous simulation was conducted to show the impact of the fumigation saturation parameter *a*. As we mentioned before, a smaller value *a* indicates a more prepared community to the increasing number of infected individuals. From the expression of *ℛ*_0_ in (15), it can be seen that *a* does not appear in *ℛ*_0_. Hence, we conclude that *a* does not impact the size of *ℛ*_0_. However, as we have shown in Figure 11, a smaller value of *a* reduces the size of total infected humans and mosquitoes in the malaria-endemic equilibrium point. Therefore, it can be concluded that although the level of community readiness to carry out fumigation does not affect the final state of population (endemic or not), it is clear that the higher the community readiness (the smaller the value of *a*), then the smaller the total size of the infected population in malaria-endemic equilibrium.

### 5.3. Effect of Different Fumigation Strategy

As we have mentioned in sensitivity analysis on *ℛ*_0_, we find that fumigation does not affect the size of *ℛ*_0_, but it can reduce the size of malaria-endemic equilibrium when fumigation intervention increases, as shown in Figure 12.

Now, we conduct our simulation with three different scenarios, based on the measured fumigation control depending on the implementation time. In the 1^st^ and the 2^nd^ scenarios, we choose *u*_2_ to be changed depending on the time interval, using the following step function:

(33) $$\begin{array}{c} u_{2}^{1^{\text{st}}\text{scenario}}=\left(\begin{array}{cc} 0.3, & t\leq 500,\\ 0.9, & 500\leq t\leq 2000,\\ 0.3, & 2000\leq t\leq 10000, \end{array}\right.\\ \;u_{2}^{2^{\text{nd}}\text{scenario}}=\left(\begin{array}{cc} 0.3, & t\leq 10,\\ 0.9, & 10\leq t\leq 1510,\\ 0.3, & 1510\leq t\leq 10000, \end{array}\right. \end{array}$$

while the 3^rd^ scenario when *u*_2_ = 0.3 for all time *t* ∈ [0, 10000]. The result is given in Figure 13. We can see from Figure 13 that when there exist two stable malaria-endemic equilibrium points, then proper fumigation intervention may change the direction of stability of the system, which in our numerical experiment is from the large endemic size into small endemic size. When the improvement of fumigation is given too early (2^nd^ scenario), then after the fumigation intervention loosened back into 0.3, then the dynamic of total infected human goes back to the large endemic size. On the other hand, when the intervention is given several times after the first implementation (1^st^ scenario), then the dynamic of total infected humans is continuously going to the small endemic equilibrium. Based on this, it is necessary to consider the time for implementing an appropriate increase in fumigation intervention so that the solution dynamics can be directed to a smaller endemic point if the bistability phenomenon appears.

## 6. Conclusions

Malaria has long been a critical health problem in various parts of the world. Every year, hundreds of millions of people are at risk of becoming infected with malaria, with the majority of cases occurring in Africa. The disease is spread due to the bite of a female Anopheles mosquito and is caused by five different types of Plasmodium. Different types of Plasmodium that infect give different symptoms/serious illness that appears in patients with malaria. Various interventions have been and are being researched, such as vaccination, treatment, vector control with fumigation, and use of insecticide-treated bed net. The high number of cases in various parts of the world until now indicates that our understanding of malaria is still not sufficient to help us optimally control the spread of malaria.

In this research, we introduce a new malaria model that considers two important factors: the use of a new treatment (tafenoquine) to prevent relapse and a saturated fumigation function. The fundamental properties, the existence and stability criteria of the equilibrium points, and how they relate to the basic reproduction number are analyzed in detail. We use Descartes's rule of signs to show a possible number of malaria-endemic equilibrium points when the basic reproduction is less or larger than one. We find that it is possible to have more than one endemic equilibrium when the basic reproduction number is larger than one. Our bifurcation analysis shows how our model consistently exhibits a forward bifurcation at the basic reproduction number equal to one. However, our numerical simulations show forward bifurcation phenomena with hysteresis. This phenomenon results in the emergence of three malaria-endemic equilibrium for a basic reproduction number larger than one.

Our sensitivity analysis shows that tafenoquine has a big potential to control the spread of malaria by preventing the possibility of exposed individuals from relapsing. Furthermore, we also find that although fumigation does not affect the basic reproduction number, it can reduce the number of infected individuals at malaria-endemic equilibrium. Furthermore, a numerical investigation on implementing a high intensity of fumigation in a short time intervention interval may lead to a final switching condition if the forward with hysteresis phenomena appears. We find that when fumigation is implemented in a proper time interval, the direction of endemic equilibrium can be “kicked down” into the smaller size of malaria-endemic equilibrium, which is easier to control with other intervention strategies. We hope that the results of our research in this article can provide another perspective in evaluating the possibility of implementing tafenoquine and fumigation in the field.

## Figures and Tables

**Figure 1:** Transmission diagram of malaria model in (7).

**Figure 2:** Histogram of normalized sensitivity analysis of *ℛ*_0._

**Figure 3:** Level set of *ℛ*_0_ with respect to *p*, *α*, and *u*_1_.

**Figure 4:** Type of bifurcation phenomena of system (7). The red figure presents *I*^†^ in *MEEE*, the blue curve is *I*^∗^ in *MFE*, and the magenta curve presents the basic reproduction number as a function of *β*_*h*_. The solid and dotted curve present stable and unstable equilibrium point, respectively.

**Figure 5:** Autonomous simulation of Figure 4(a): trajectories of infected compartments for many different initial conditions toward MFE when *ℛ*_0_ = 0.98 < 1. The left figure is simulation for the first 300 days, while the right figure is simulation for days 95000 to 100000.

**Figure 6:** Autonomous simulation of Figure 4(a): trajectories of infected compartments for many different initial conditions toward MEE when *ℛ*_0_ = 4.902 > 1. The left figure is simulation for 300 days, while the right figure is simulation for days 95000 to 100000.

**Figure 7:** Autonomous simulation of Figure 4(b): trajectories of infected compartments for many different initial conditions toward single *MEE* when *ℛ*_0_ = 1.225 > 1. The left figure is simulation for 300 days, while the right figure is simulation for days 95000 to 100000.

**Figure 8:** Autonomous simulation of Figure 4(b): trajectories of infected compartments for many different initial conditions toward two stable *MEE* when *ℛ*_0_ = 3.6769 > 1, depending on the initial conditions. The left figure is simulation for 300 days, while the right figure is simulation for days 95000 to 100000.

**Figure 9:** The bifurcation diagram of system (7) depends on the value of fumigation rate. We use the same parameter values for each curve, except *u*_2_ = 0 (black), *u*_2_ = 0.1 (magenta), *u*_2_ = 0.2 (green), *u*_2_ = 0.3 (red), and *u*_2_ = 0.4 (cyan)

**Figure 10:** Simulations showing the effect of vector-bias parameter (*α*) on the total of infected human (left) and mosquitoes (right). We use same parameter values as in Table 2, except *u*_1_ = 0.1, *u*_2_ = 0.05, *p* = 0.8, and *α* varying: *α* = 5 (black), *α* = 4 (red), *α* = 3 (green), *α* = 2 (blue), and *α* = 1 (cyan).

**Figure 11:** Simulations showing the effect of fumigation saturation parameter (*a*) on the total of infected human (left) and mosquitoes (right). We use same parameter values as in Table 2, except *u*_1_ = 0.1, *u*_2_ = 0.2, *p* = 0.8, and *a* varying: *a* = 20 (blue), *a* = 50 (green), *a* = 100 (red), *a* = 200 (cyan), and *a* = 300 (black). With this set of parameter, we have that *ℛ*_0_ = 1.23.

**Figure 12:** Effect of fumigation on the endemic size of total infected human (left) and mosquitoes (right). Three different values of *u*_2_ are given: 0 (red), 0.5 (blue), and 1 (green) do not change the value of *ℛ*_0_, which is always 1.77.

**Figure 13:** Simulations on the total infected human showing the effect of early (green), late (red), and no change (blue) of fumigation intervention.

**Table 1:** Biological interpretation of parameters in system (7).

Par	Description	Dimension	Value	Ref.
*Λ*_*h*_	Number of newborn in human per day	Human/Day	1000/65 × 365	[15]
*Λ*_*v*_	Number of newborn in mosquitoes per day	Mosquitoes/Day	1000/21	[15]
*β*_*h*_	Infection rate of mosquito to human	1/Mosquito × day	0.022	[30, 31]
*β*_*v*_	Infection rate of human to mosquito	1/Human × day	0.24	[30, 31]
*α*	Vector-bias coefficient	—	4	[32]
*u*_1_	Rate of treatment with tafenoquine	1/Day	[0,1]	Assumed
*u*_2_	Vector control with fumigation	1/Day	[0,1]	Assumed
*μ*_*h*_	Natural death rate of human	1/Day	1/65 × 365	[15]
*μ*_*v*_	Natural death rate of mosquito	1/Day	1/21	[30]
*η*	Natural incubation rate	1/day	0.0833	[18]
*p*	Proportion of treated individual who succeeds in treatment	—	0.8	Assumed
*δ*	Incubation rate due to use of tafenoquine	1/Day	0.016	Assumed
*κ*	Recovery rate tafenoquine treatment	1/Day	0.0166	Assumed
*γ*	Recovery rate	1/Day	0.0035	[30]
*a*	Saturation coefficient of fumigation	Human	10	Assumed
*ξ*	Waning rate of temporal immunity	1/Day	0.005	[33]

**Table 2:** Normalized sensitivity indices of *ℛ*_0_ with respect to *β*_*h*_, *β*_*v*_, *α*, *u*_1_, *u*_2_, *η*, *δ*, *p*, *κ*, *γ*, *ξ*, and *a*.

Par (*ρ*)	Γ_*ρ*_^*ℛ*_0_^	Par (*ρ*)	Γ_*ρ*_^*ℛ*_0_^	Par (*ρ*)	Γ_*ρ*_^*ℛ*_0_^
*β*_*h*_	0.5	*β*_*v*_	0.5	*α*	0.5
*u*_1_	-0.191	*u*_2_	0	*η*	0.191
*δ*	0.129	*p*	−0.6477	*κ*	-0.120
*γ*	-0.494	*ξ*	0	*a*	0

**Table 3:** Possible number of positive roots of polynomial *G*(*Ω*, *I*), when *ℛ*_0_ > 1.

Case	*k*_6_	*k*_5_	*k*_4_	*k*_3_	*k*_2_	*k*_1_	*k*_0_	Possible positive roots
1	—	+	+	+	+	+	+	1
2	—	+	+	+	+	—	+	1 or 3
3	—	+	+	+	—	+	+	1 or 3
4	—	+	+	+	—	—	+	1 or 3
5	—	+	+	—	+	+	+	1 or 3
6	—	+	+	—	+	—	+	1, 3, or 5
7	—	+	+	—	—	+	+	1 or 3
8	—	+	+	—	—	—	+	1 or 3
9	—	+	—	+	+	+	+	1 or 3
10	—	+	—	+	+	—	+	1, 3, or 5
11	—	+	—	+	—	+	+	1, 3, or 5
12	—	+	—	+	—	—	+	1, 3, or 5
13	—	+	—	—	+	+	+	1 or 3
14	—	+	—	—	+	—	+	1, 3, or 5
15	—	+	—	—	—	+	+	1 or 3
16	—	+	—	—	—	—	+	1 or 3
17	—	—	+	+	+	+	+	1
18	—	—	+	+	+	—	+	1 or 3
19	—	—	+	+	—	+	+	1 or 3
20	—	—	+	+	—	—	+	1 or 3
21	—	—	+	—	+	+	+	1 or 3
22	—	—	+	—	+	—	+	1, 3, or 5
23	—	—	+	—	—	+	+	1 or 3
24	—	—	+	—	—	—	+	1 or 3
25	—	—	—	+	+	+	+	1
26	—	—	—	+	+	—	+	1 or 3
27	—	—	—	+	—	+	+	1 or 3
28	—	—	—	+	—	—	+	1 or 3
29	—	—	—	—	+	+	+	1
30	—	—	—	—	+	—	+	1 or 3
31	—	—	—	—	—	+	+	1
32	—	—	—	—	—	—	+	1

**Table 4:** Possible number of positive roots of polynomial *G*(*Ω*, *I*), when *ℛ*_0_ < 1.

Case	*k*_6_	*k*_5_	*k*_4_	*k*_3_	*k*_2_	*k*_1_	*k*_0_	Possible positive roots
33	—	+	+	+	+	+	—	0 or 2
34	—	+	+	+	+	—	—	0 or 2
35	—	+	+	+	—	+	—	0, 2, or 4
36	—	+	+	+	—	—	—	0 or 2
37	—	+	+	—	+	+	—	0, 2, or 4
38	—	+	+	—	+	—	—	0, 2, or 4
39	—	+	+	—	—	+	—	0, 2, or 4
40	—	+	+	—	—	—	—	0 or 2
41	—	+	—	+	+	+	—	0, 2, or 4
42	—	+	—	+	+	—	—	0, 2, or 4
43	—	+	—	+	—	+	—	0, 2, 4, or 6
44	—	+	—	+	—	—	—	0, 2, or 4
45	—	+	—	—	+	+	—	0, 2, or 4
46	—	+	—	—	+	—	—	0, 2, or 4
47	—	+	—	—	—	+	—	0, 2, or 4
48	—	+	—	—	—	—	—	0 or 2
49	—	—	+	+	+	+	—	0 or 2
50	—	—	+	+	+	—	—	0 or 2
51	—	—	+	+	—	+	—	0, 2, or 4
52	—	—	+	+	—	—	—	0 or 2
53	—	—	+	—	+	+	—	0, 2, or 4
54	—	—	+	—	+	—	—	0, 2, or 4
55	—	—	+	—	—	+	—	0, 2, or 4
56	—	—	+	—	—	—	—	0 or 2
57	—	—	—	+	+	+	—	0 or 2
58	—	—	—	+	+	—	—	0 or 2
59	—	—	—	+	—	+	—	0, 2, or 4
60	—	—	—	+	—	—	—	0 or 2
61	—	—	—	—	+	+	—	0 or 2
62	—	—	—	—	+	—	—	0 or 2
63	—	—	—	—	—	+	—	0 or 2
64	—	—	—	—	—	—	—	0

## Data Availability

No data were used to support this study.

## Appendix

### A. Proof of Theorem 1

We proof our theorem by analyzing the behaviour of each variables on it boundary planes. From malaria model in system (7), we have the dynamics on the boundary of ℝ_+_^7^ as follows.

(A.1) $$\begin{array}{c} {\left.\frac{dS}{dt}\right|}_{S=0,E\geq 0,T\geq 0,I\geq 0,R\geq 0,U\geq 0,W\geq 0}=\Lambda_{h}>0,\\ {\left.\frac{dE}{dt}\right|}_{S\geq 0,E=0,T\geq 0,I\geq 0,R\geq 0,U\geq 0,W\geq 0}=\beta_{h}W\frac{S}{S+E+T+\alpha I+R}\geq 0,\\ {\left.\frac{dT}{dt}\right|}_{S\geq 0,E\geq 0,T=0,I\geq 0,R\geq 0,U\geq 0,W\geq 0}=u_{1}E\geq 0,\\ {\left.\frac{dI}{dt}\right|}_{S\geq 0,E\geq 0,T\geq 0,I=0,R\geq 0,U\geq 0,W\geq 0}=\left(1-p\right)\delta T+\eta E\geq 0,\\ {\left.\frac{dR}{dt}\right|}_{S\geq 0,E\geq 0,T\geq 0,I\geq 0,R=0,U\geq 0,W\geq 0}=p\kappa T+\gamma I\geq 0,\\ {\left.\frac{dU}{dt}\right|}_{S\geq 0,E\geq 0,T\geq 0,I\geq 0,R\geq 0,U=0,W\geq 0}=\Lambda_{v}>0,\\ {\left.\frac{dW}{dt}\right|}_{S\geq 0,E=0,T\geq 0,I\geq 0,R\geq 0,U\geq 0,W=0}=\beta_{h}W\frac{S}{S+E+T+\alpha I+R}\geq 0. \end{array}$$

It can be seen that all the rates of variables are nonnegative on the boundary of ℝ_+_^7^. Therefore, if we start in the interior of the nonnegative *𝒟*, we shall always remain in this region in view that the direction of the vector field is inward on the boundary planes. Thus, the nonnegativity of all solutions of system (7) is guaranteed.

Next, we continue to show the uniqueness solution of system (7) by showing the boundedness of *N*_*h*_ and *N*_*v*_. Adding the first five equations in system (7) together, we get

(A.2) $$\begin{array}{c} \frac{dN_{h}\left(t\right)}{dt}=\Lambda_{h}-\mu_{h}\left(S+E+T+I+R\right),=\Lambda_{h}-\mu_{h}N_{h}. \end{array}$$

Solving the above differential equations with respect to *N*_*h*_(*t*) and with a positive initial condition *N*_*h*_(0) > 0 gives

(A.3) $$\begin{array}{c} N_{h}\left(t\right)=N_{h}\left(0\right)\exp\left(-\mu_{h}t\right)+\frac{\Lambda_{h}}{\mu_{h}}. \end{array}$$

Hence, if we take *t*⟶∞, then we have that *N*_*h*_(*t*) is eventually bounded by *Λ*_*h*_/*μ*_*h*_. To be precise, we have that the biological feasible region of human population of system (7) is

(A.4) $$\begin{array}{c} 0\leq S+E+T+I+R\leq \frac{\Lambda_{h}}{\mu_{h}}. \end{array}$$

For mosquito population, by adding the last two equation in system (7), we have

(A.5) $$\begin{array}{c} \frac{dN_{v}\left(t\right)}{dt}=\Lambda_{v}-\left(\mu_{v}+u_{2}\frac{I}{a+I^{2}}\right)\left(U\left(t\right)+W\left(t\right)\right),\\ =\Lambda_{v}-\left(\mu_{v}+u_{2}\frac{I}{a+I^{2}}\right)N_{v}\left(t\right),\\ <\Lambda_{v}-\mu_{v}N_{v}\left(t\right). \end{array}$$

Solving the above expression with respect to *N*_*v*_(*t*) and with positive initial condition *N*_*v*_(0) > 0, we get

(A.6) $$\begin{array}{c} N_{v}\left(t\right)<N_{v}\left(0\right)\exp\left(-\mu_{v}t\right)+\frac{\Lambda_{v}}{\mu_{v}}. \end{array}$$

Hence, if we take *t*⟶∞, we have that *N*_*v*_(*t*) is eventually bounded by *Λ*_*v*_/*μ*_*v*_. Hence, the biological feasible region of mosquito population is

(A.7) $$\begin{array}{c} 0\leq U+W\leq \frac{\Lambda_{v}}{\mu_{v}}. \end{array}$$

Hence, the proof is complete.

### B. Possible Positive Root of Polynomial (7) when *ℛ*_0_ > 1

For an example, substitute parameter values as in Figure 4(b) and *β*_*h*_ = 0.0015 to polynomial *G*(*Ω*, *I*) in (19), we have

(B.1) $$\begin{array}{c} G\left(I\right)=-2.3\times 10^{-17}I^{6}-1.2\times 10^{-14}I^{5}+8.3\times 10^{-13}I^{4}-4.5\times 10^{-12}I^{3}+3.9\times 10^{-12}I^{2}-4.3\times 10^{-11}I+9.01\times 10^{-11}, \end{array}$$

which is the case number 22. Solve *G*(*I*) = 0 with respect to *I*, and then, we have 3 positive roots of *I*, i.e., 1.91, 6.23, and 53.6.

### C. Possible Positive Root of Polynomial (7) when *ℛ*_0_ < 1

For an example, substituting parameter values as in Figure 4(a) and *β*_*h*_ = 0.0002 to polynomial *G*(*Ω*, *I*) in (19), we have

(C.1) $$\begin{array}{c} G\left(I\right)=-2.3\times 10^{-17}I^{6}-9.3\times 10^{-15}I^{5}-1.9\times 10^{-13}I^{4}-7.4\times 10^{-12}I^{3}-1.4\times 10^{-10}I^{2}-1.4\times 10^{-9}I-2.7\times 10^{-8}, \end{array}$$

which is the case number 64. Solve *G*(*I*) = 0 with respect to *I*, and then, we have no positive roots.

### D. Expression of *𝒜*

(D.1)
$$\begin{array}{c} A=A_{1}+A_{2}, \end{array}$$

where

(D.2) $$\begin{array}{c} A_{1}=-m_{1}2{\left(\eta \mu_{h}+\delta \left(u_{1}+\eta \right)\left(1-p\right)+\eta p\kappa \right)}^{2}\left[\mu_{h}^{3}+\left(\delta \left(1-p\right)+p\kappa +\eta \alpha +\xi +u_{1}+\gamma_{1}\right)\mu_{h}^{2}\cdots \right.+\left(\left(\eta \alpha +\alpha u_{1}+\xi +\gamma_{1}\right)\left(1-p\right)\delta +p\kappa \left(\eta \alpha +\xi +\gamma_{1}+u_{1}\right)+\gamma_{1}\left(\xi +\eta +u_{1}\right)+\xi \left(\eta \alpha +u_{1}\right)\right)\mu_{h}\cdots +\left(\left(\xi +\eta +u_{1}\right)\gamma_{1}+\xi \alpha \left(\eta +u_{1}\right)\right)\left(1-p\right)\delta +\kappa \left(\left(\xi +\eta +u_{1}\right)\gamma_{1}+\xi \eta \alpha \right)p+\gamma_{1}\xi u_{1},\\ A_{2}=-\frac{1}{\Lambda_{v}\alpha \beta_{v}\mu_{h}\delta \left(1-p\right)}\left[\left(\gamma_{1}+\mu_{h}\right)\Lambda_{h}\mu_{v}\left(\left(1-p\right)\delta +p\kappa +\mu_{h}\right)\left(\frac{\beta_{v}\Lambda_{v}\alpha \mu_{h}^{2}}{{\left(\gamma_{1}+\mu_{h}\right)}^{2}u_{1}^{2}\Lambda_{h}^{2}\left(\mu_{h}+\xi \right)\mu_{v}}\left(2m_{2}m_{3}\right)+\frac{2\left(\delta \left(1-p\right)+p\kappa +\mu_{h}\right)\left(\delta \left(\eta +u_{1}\right)\left(1-p\right)+\eta \left(p\kappa +\mu_{h}\right)\right)\beta_{v}\Lambda_{v}\alpha \mu_{h}^{2}}{u_{1}^{2}\Lambda_{h}^{2}\mu_{v}\left(\gamma_{1}+\mu_{h}\right)}\cdots +\frac{2\left(\delta \left(\eta +u_{1}\right)\left(1-p\right)+\eta \left(\kappa p+\mu_{h}\right)\right)\beta_{v}\Lambda_{v}\alpha \mu_{h}^{2}}{\left(\gamma_{1}+\mu_{h}\right)u_{1}n\mu_{v}\Lambda_{h}^{2}}\cdots +\frac{2\left(\delta \left(\eta +u_{1}\right)\left(1-p\right)+\eta \left(\kappa p+\mu_{h}\right)\right)\left(\delta \gamma_{1}\left(\eta +u_{1}\right)\left(1-p\right)+\kappa p\gamma_{1}\left(\eta +u_{1}\right)\kappa p\mu_{h}u_{1}+\eta \gamma_{1}\mu_{h}\right)\beta_{v}\Lambda_{v}\alpha \mu_{h}^{2}}{{\left(\gamma_{1}+\mu_{h}\right)}^{2}u_{1}^{2}\left(\mu_{h}+\xi \right)\mu_{v}\Lambda_{h}^{2}}\cdots +\frac{2\left(\delta \left(\eta +u_{1}\right)\left(1-p\right)+\eta \left(\kappa p+\mu_{h}\right)\right)\left(\alpha a\beta_{v}\mu_{h}+u_{2}\Lambda_{h}\right)\left(\left(1-p\right)\left(\eta +u_{1}\right)\delta +\eta \left(p\kappa +\mu_{h}\right)\right)\Lambda_{v}\beta_{v}\alpha \mu_{h}}{{\left(\gamma_{1}+\mu_{h}\right)}^{2}u_{1}^{2}a\Lambda_{h}^{2}\mu_{v}^{2}}\cdots +\frac{2\left(\delta \left(\eta +u_{1}\right)\left(1-p\right)+\eta \left(\kappa p+\mu_{h}\right)\right)\Lambda_{v}\alpha \beta_{v}\mu_{h}u_{2}\left(\delta \left(1-p\right)\left(\eta +u_{1}\right)+\eta \left(p\kappa +\mu_{h}\right)\right)}{{\left(\gamma_{1}+\mu_{h}\right)}^{2}u_{1}^{2}\Lambda_{h}\mu_{v}^{2}a}\cdots +\frac{2\left(\delta \left(\eta +u_{1}\right)\left(1-p\right)+\eta \left(\kappa p+\mu_{h}\right)\right)\beta_{v}\Lambda_{v}\alpha^{2}\mu_{h}^{2}}{\left(\gamma_{1}+\mu_{h}\right)u_{1}\mu_{v}\Lambda_{h}^{2}}\right)\right], \end{array}$$

with

(D.3) $$\begin{array}{c} m_{1}=\frac{1}{\delta u_{1}^{2}\Lambda_{h}^{2}\mu_{v}^{2}\left(1-p\right)\left(u_{1}+\eta +\mu_{h}\right){\left(\gamma_{1}+\mu_{h}\right)}^{2}\left(\mu_{h}+\xi \right)},\\ m_{2}=\mu_{h}^{3}+\left(\left(1-p\right)\delta +p\kappa +\xi +\eta +\gamma_{1}+u_{1}\right)\mu_{h}^{2}\cdots \left(\left(\xi +\eta +\gamma_{1}+u_{1}\right)\left(1-p\right)\delta +\kappa \left(\xi +\eta +\gamma_{1}+u_{1}\right)p+\left(\xi +\eta +u_{1}\right)\gamma +\xi \left(\eta +u_{1}\right)\right)\mu_{h}+\cdots \left(1-p\right)\left(\left(\xi +\eta +u_{1}\right)\gamma_{1}+\xi \left(\eta +u_{1}\right)\right)\delta +\kappa \left(\left(\xi +\eta +u_{1}\right)\gamma_{1}+\eta \xi \right)p+\gamma_{1}\xi u_{1},\\ m_{3}=\left(\delta \left(\eta +u_{1}\right)\left(1-p\right)+\eta \kappa p+\eta \mu_{h}\right). \end{array}$$

Since *𝒜*_1_ and *𝒜*_2_ are negative, then we have *𝒜* < 0.
